# Mechanism of High-Tech Enterprises' Technological Practices Affected by the Split Fault of Knowledge Innovation Network

**DOI:** 10.1155/2022/2984136

**Published:** 2022-05-13

**Authors:** JianLin Yuan, Yue Pan, Qilei Jiang

**Affiliations:** College of Management, Liaoning University of Technology, Jinzhou 121001, China

## Abstract

Knowledge innovation ability is the source of value realization of high-tech enterprises, and the acquisition of high-value knowledge is important. Taking knowledge as the intermediary variable, knowledge field activity and knowledge fermentation as mediating variables, and knowledge mobilization and knowledge network position transition as moderating variables, the conceptual model and theoretical analysis framework of the impact mechanism of knowledge innovation network fragmentation fault on technology practices is constructed and the moderated mediating effect model is derived. Taking high-tech enterprises as empirical samples, 538 valid questionnaires were obtained online and offline and the nonpercentile bootstrap method based on deviation correction was used to empirically investigate the influence mechanism and transmission path of knowledge innovation network fragmentation fault on high-tech enterprises' technological practices. The empirical results show that the main effect of knowledge innovation network fragmentation fault on high-tech enterprise technology practices is significant. Knowledge field activity and knowledge fermentation play a differential mediating role in knowledge innovation network split fault and Technology Convention. Knowledge field activity and knowledge fermentation play a partial mediating role in knowledge innovation network split fault and Technology Convention. Knowledge mobilization partially moderates the split fault of knowledge innovation network and technological practices. Knowledge mobilization positively moderates the positive effect of split fault of knowledge innovation network on technological practices and significantly positively moderates the mediating effect of knowledge field activity and knowledge fermentation, resulting in the moderated mediating effect. Knowledge network location transition plays a part of moderating role in knowledge innovation network split fault and Technology Convention. Knowledge network location transition positively moderates the positive impact of knowledge innovation network split fault on Technology Convention and significantly positively moderates the mediating role of knowledge field activity and knowledge fermentation, resulting in a moderated mediating effect. Knowledge innovation network split fault, knowledge field activity and knowledge fermentation, knowledge mobilization and knowledge network location transition, and the combination of technological practices can be the antecedents of promoting technological practices in high-tech enterprises. Through the research on the mechanism of knowledge innovation network split fault in the technological practices of high-tech enterprises, the connotation of knowledge innovation network split fault is enriched, the influencing factors of technological practices are clarified, and the value-added knowledge is promoted and has guiding and reference significance for the innovation knowledge acquisition and competitiveness improvement of high-tech enterprises.

## 1. Introduction

In 2019, COVID-19 will not only seriously threaten the health of the masses but also hit the world economic development. Hitherto unknown, the world has spared no effort to develop a vaccine for COVID-19 against human diseases, such as manpower, material resources, and funds. In less than a year, the new crown antibody vaccine has provided a reliable material foundation for the global fight against COVID-19. This is a successful example of human being's technology and science. The world is changed by knowledge, and the future is created by technology. Productivity is changed by science and technology. That is proved by the history of human development. Obtaining technological breakthroughs and ensuring the continuous growth of scientific and technological strength are not only the source of long-term competitiveness of different countries but also an issue that scholars all over the world strive to explore.

The competition limited to a single technological innovation activity has been difficult to meet the needs of modern scientific and technological progress. The integrated, systematic, and networked competition pattern has become an inevitable development trend. The networking of knowledge innovation is a common concern of scholars in recent years, and it is also the development strategy of high-tech enterprises in various countries [1]. Based on the innovation network, high-tech enterprises reconstruct the knowledge technology system, break through the technical barriers of knowledge integration, fully optimize the organizational structure, give full play to the leading advantages of industry technology, and obtain the voice of technological competition in the spirit of “sales generation-development generation-design generation” [2].

Enterprise technical practices are the technical criterion and paradigms that it can serve the competitive needs of enterprises, and those is based on innovative technology, adhering to innovative thinking and adhering to enterprise technical norms. The enterprise technology boundary is broken by the continuous evolution of knowledge innovation network and breaks the enterprise organization reconstructed, which promotes the mutation of enterprise technology practice, improves the overall technical level of enterprises, and helps enterprises innovate and compete. The split fault of knowledge innovation network is a process that itself originates from external changes and internal structure reorganization and constantly deepens self-adaptation. The split fault of knowledge innovation network strengthens the existing technical norms of high-tech enterprises, forms new technical practices, and promotes the technological progress of high-tech enterprises. The evolution process of the split fault of knowledge innovation network has made an interpretation of the technical practices of high-tech enterprises to a certain extent, but it can be still studied to strengthen its value. Firstly, in the evolution process of knowledge innovation network splitting fault, it will be affected by “field strength,” that is, the activity of knowledge field [3]. The gravity around knowledge innovation network directly determines the stability of its network and the evolution direction of its division, which brings great changes to the technical practices of high-tech enterprises. The nodes in the links of the knowledge innovation network are directly related to the number and quality of the split faults of the innovation network. The extension and mutation of the knowledge chain will affect the overall structure of the knowledge innovation network and the standardization of the technical practices of high-tech enterprises [4]. Secondly, the activity of the internal nodes of the knowledge innovation network affects the progress of the division fault of high-tech enterprises. Through the changes of the internal knowledge nodes of the high-tech enterprise network, it can effectively stimulate the endogenous driving force of the knowledge innovation network and create the normative change of the technical practices of high-tech enterprises. The changing of the external mechanism of knowledge innovation network can squeeze the stability of its internal structure, trigger its knowledge gene mutation, produce a spillover effect, and then break the original model and change the technical practice of high-tech enterprises. Finally, Kang and Liu studied the split fault of knowledge innovation network and had a clear understanding of the change of technical practice triggered by the split fault of knowledge innovation network, but the impact mechanism of the split fault of knowledge innovation network on technical practice needs to be further deepened [5].

To sum up, from the perspective of technological innovation network, this study establishes a theoretical model of the impact path of knowledge split fault innovation network on technological practices, takes knowledge field activity and knowledge fermentation as intermediary variables, and takes knowledge mobilization and knowledge network location transition as regulatory variables to reveal the impact mechanism of knowledge split fault on technological practices. It provides a reference for enterprises to efficiently and continuously obtain benefits from innovation and also provides theoretical support for expanding the research of technical practices.

## 2. Theoretical Basis and Research Hypothesis of the Relevant Literature

### 2.1. Knowledge Innovation Network Split Fault and Technical Practices

The split fault of knowledge innovation network is the evolution process of knowledge system adapting to the changes of internal and external environment. Referring to the relevant concepts of geography and based on the spatial position relationship between fault strike and fold axis, the split fault of knowledge innovation network is divided into vertical fault of knowledge innovation network, horizontal fault of knowledge innovation network, and oblique fault of knowledge innovation network (as shown in Figure 1). Corsaro et al. and Andrew et al. attributed the division of knowledge innovation network to the pressure given by the external environment [6, 7]. Dang et al. believe that the horizontal fault of knowledge innovation network is the mutual cooperation and collision of homogeneous enterprises, forming the gene variation of enterprise knowledge innovation network and constructing new systems and subgroups [8]. Lau and Murnighan believe that the vertical fault of knowledge innovation network is the gene mutation of enterprise knowledge innovation network formed by the complementary and impact of knowledge generated by the cooperation between upstream and downstream enterprises, which evolved into a new knowledge network system [9]. Heidl et al. and Wu and Li believe that the split fault of knowledge innovation network is the result of the joint action of multiple factors; that is, homogeneous enterprises cooperate, complement, and collide with each other, and it is also an oblique fault knowledge innovation network system formed by mutual learning, discussion, and conflict between different types of enterprises [10, 11].

Li and Hambrick believe that, in the process of continuous differentiation and evolution of knowledge innovation network splitting fault, subgroup is the core of knowledge innovation network splitting fault [12]. Homogeneous and heterogeneous enterprises cooperate and complement each other, produce the replacement of knowledge content, act on the knowledge carrier, make qualitative changes, update the technical norms and norms of high-tech enterprises, and improve the level of technical practices. Dagnino et al. believed that the knowledge gene of knowledge innovation split fault is the source of mutation [13]. The polarization of the external environment triggers the split fault of knowledge innovation and the variation of internal genes and generates new knowledge factors so as to derive new knowledge system, change the original technical standards of enterprises, and accelerate the upgrading of enterprise technical practices.

Mutual cooperation and complementarity among enterprises accelerate the replacement and innovation of enterprise knowledge content. The differences in mechanism, style, trust, distance, and concept in interenterprise cooperation cause the division and fault of knowledge innovation network, change the original operation mode and technical standards, and upgrade the technical practice [14]. Enterprises choose to cooperate with individuals with their own cultural similarity and mutual technological complementarity. In mutual cooperation, there are both input and output, and the strength of partnership will deepen [15, 16]. The strengthening of the depth of cooperation will bring rapid knowledge mobility, improve the speed of knowledge renewal, accelerate the split fault of knowledge innovation, differentiate more and more subgroups, and form new technical models, and the original technical practices will be replaced.

To sum up, the split fault of knowledge network innovation is the result of mutual integration, exchange, complementarity, and collision of knowledge among enterprises. The change of knowledge content accelerates the formation of new knowledge subgroups, evolves new technical specifications, breaks the original technical standards of enterprises, and forms new technical practices. Based on this, a hypothesis is put forward.

H1: the split fault of knowledge innovation network has a positive impact on technological inertia.

### 2.2. Activity of Knowledge Field and Intermediary Role of Knowledge Fermentation

#### 2.2.1. Intermediary Role of Knowledge Field Activity

Referring to the concept of electromagnetic field in physics, Nonaka and Takeuchi clearly expound on the connotation of knowledge field and points out that knowledge field is a spatial framework gathered by a series of entities in the process of knowledge differentiation, derivation, migration, and diffusion [17]. In this spatial system, all subjects maintain activity, blend, cooperate, collide, embed, and iterate with each other so as to achieve the sublimation of knowledge value. The activity of knowledge field depends on the dynamics of knowledge genes [18], the mobility of knowledge genes [19], and the degree of integration with internal and external knowledge determines the changing level of knowledge connotation and affects the split level of knowledge innovation network.

The enrichment of knowledge determines the strength of knowledge field, and the strength of knowledge field determines the dynamics of knowledge gene. High-tech enterprises and other enterprises can effectively cooperate and cooperate with each other, which makes it easier to promote the mutual integration and replacement of knowledge, enhance the ability of enterprise knowledge innovation, intensify the division and fault of knowledge innovation network, and accelerate the change of enterprise technical practices. Gan and Qi and others believe that the activity of knowledge field is determined by the activity and openness of knowledge field, which has the characteristics of dual attributes [20]. The high activity of knowledge field means that the gene vitality in the knowledge field is vigorous, which means that the content of enterprise knowledge is rich and the ability of knowledge derivation is strong. The openness of the knowledge field is strong [21]; that is, the exchange, integration, and overlap of internal knowledge and external knowledge in the field have high intensity, and there is also frequent and in-depth communication between enterprises and external knowledge. Zhao believes that, in addition to the field strength affecting its activity, the “knowledge potential” difference formed by the differences of individual knowledge in the field can also stimulate the activity of knowledge genes in the field, aggravate the embedding and overflow of knowledge connotation, constantly expand the split fault of knowledge innovation network, and accelerate the renewal of enterprise technical practices [22].

To sum up, the activity of knowledge field can accelerate the activity of knowledge gene, promote the continuous evolution, expansion, extension, and sublimation of knowledge connotation, the continuous upgrading, and updating of knowledge content, accelerate the updating and iteration of the split fault of knowledge innovation network, promote the generation of enterprise technical specifications and standards, and change the original technical practices of enterprises. Therefore, assumptions are put forward.

H2: knowledge field activity plays an intermediary role in the positive effect of knowledge network splitting fault on enterprise technology practice.

#### 2.2.2. Intermediary Role of Knowledge Fermentation

Barthelme et al. studied the feasibility of knowledge evolution in view of the principle of bionics [23]. On this basis, He put forward the concept of knowledge fermentation [24]. He compared knowledge growth with the biological fermentation process and proposed that knowledge fermentation is a process of qualitative change based on knowledge genes and cultivated by a certain knowledge matrix under the action of knowledge enzymes in a suitable growth environment [25–27] (Figure 2). The essence of knowledge innovation is the process of knowledge transfer, growth, embedding, and derivation. Li and Zhang divide it into four different stages, that is, the process from tacit knowledge to explicit knowledge and then to tacit knowledge, that is, knowledge socialization, knowledge externalization, knowledge combination, and knowledge internalization [28]. The process of knowledge returning from recessive to recessive is not a simple copy and superposition, but a process of knowledge reorganization, combination, and sublimation. This process strengthens the upgrading of knowledge connotation, strengthens the bone, strengthens the physique, and takes on a new look.

Knowledge genes derived from knowledge matrix (knowledge source, which can be regarded as enterprise innovation network), through knowledge enzyme (knowledge coordination and management mechanism), under a certain knowledge growth environment (knowledge exchange and knowledge fusion), converge in the knowledge fermentation bar through a certain carrier (knowledge transmission and knowledge transfer), from quantitative change to qualitative change, in a certain specific spatial system. Knowledge has been sublimated and transformed, the number of knowledge innovation network split faults has increased sharply, breaking the original knowledge norms and standards, new technical norms and standards have emerged from time to time, and technical practices have been upgraded [29–32].

To sum up, knowledge fermentation can accelerate the mutation of knowledge genes, enhance knowledge connotation, and constantly expand knowledge content in cooperation with the external environment. The collection of knowledge content in the knowledge fermentation bar accelerates the upgrading of knowledge itself, promotes the renewal and iteration of the split layer of knowledge innovation network, and promotes the generation of enterprise technical specifications and standards, changing the original technical practices of the enterprise. Therefore, assumptions are put forward.

H3: knowledge fermentation plays an intermediary role in the positive effect of knowledge network fragmentation on enterprise technology practices.

### 2.3. The Regulatory Role of Knowledge Mobilization and Knowledge Network Position Transition

#### 2.3.1. Regulatory Role of Knowledge Mobilization

The concept of knowledge mobilization comes from Canada [33]. Shields et al. further enriched it and pointed out that knowledge mobilization multiplies knowledge integration [34]. Yao and Tong deeply analyzed the connotation and performance dimensions of knowledge mobilization and pointed out that knowledge mobilization is a continuous flowing process composed of knowledge collection, knowledge identification, and knowledge transfer based on the specific objectives of the organization [35]. Through its strong endogenous power, knowledge mobilization searches for relevant information inside and outside the system, carries out effective combination, translation, and screening, eliminates the rough, extracts the fine, eliminates the false and retains the true, and then condenses and sublimates the collected knowledge to achieve the purpose of innovation [36]. In this process, on the one hand, its integration ability is outstanding and strong, and it can encode and classify different systems, scattered and professional knowledge translation, transformation, breaking down knowledge barriers, and identifying and accepting demanders. On the other hand, knowledge mobilization has good fecundity, constantly pushing through the old and bringing forth the new, breaking the original pattern of knowledge, effectively eliminating the stickiness of knowledge [37], collecting relevant knowledge content, transforming it, constantly splitting it, increasing the activity of knowledge, improving the activity of knowledge field, continuously creating new knowledge connotation and systems, breaking the original technical practices and accelerating the renewal of knowledge, and building new technical specifications and standards.

Knowledge mobilization from knowledge traversal to knowledge innovation is not an overnight task, but a complex process, from simple knowledge collection to knowledge extraction. This process can be divided into three different forms [38]: (1) Linear process: it is a direct transition from theoretical knowledge to practical knowledge, emphasizing the application of knowledge, and the transmission of knowledge is like a straight line. (2) Spiral process: this process emphasizes the evolution and innovation of knowledge, which is the process of constantly carrying, sorting, summarizing, sublimating, and reengineering knowledge in the search and concentration of knowledge until it meets the needs of the ultimate knowledge and emphasizes the function of knowledge reengineering. (3) Composite process: in the process of knowledge transmission, it is not a single movement process, but a complex movement experience. This process is always intertwined with the linear and spiral forms around the needs of customers so as to jointly promote the transmission and transfer of knowledge. The three knowledge channels are different, but at the same time, they all pay attention to the realization of the value of knowledge. This process is also a process of accelerating, progressive, and evolving knowledge fermentation to promote the realization of technical practices. Based on the above analysis, assumptions are put forward.

H4: knowledge mobilization positively regulates the impact of knowledge field activity and knowledge fermentation on technical inertia; that is, the higher the level of knowledge mobilization, the stronger the impact of knowledge field activity and knowledge fermentation on technical inertia.

#### 2.3.2. Regulatory Role of Knowledge Network Location Transition

The location transition of knowledge network refers to the process of knowledge migration from low level to high level in the overall network [39]. The process of position transition of knowledge network is essentially the process of energy conversion. Knowledge enriches and improves its own content through reorganization, embedding, and absorption so as to achieve the purpose of position transition. This process is also the process of transformation from kinetic energy to potential energy. This process is accompanied by the growth of knowledge potential energy, the enhancement of knowledge integration, the breakthrough of knowledge cooperation in the knowledge matrix, the acceleration of knowledge fermentation process, the breaking of the original technical barriers, the emergence of new technical specifications, and the reorganization of technical practices. Zaheer and Bell concluded that the location transition of knowledge network strengthens the epidemic resistance of knowledge gene and can effectively screen external relevant knowledge information, select knowledge content suitable for the subject to give play to its competitive advantage, and improve knowledge connotation, which is the process of continuous recombination of knowledge itself [40]. There are two main ways of knowledge network location transition: (1) Communication with the outside to obtain knowledge location transition [41]. Exchange knowledge with external systems, strengthen the connotation of their own knowledge, improve their knowledge abundance, promote their own health, and enable them to obtain sufficient energy, convert kinetic energy into potential energy, and move position so as to make a transition. (2) Knowledge internal running in to obtain knowledge position transition [42]. The external environment is not suitable for them to obtain sufficient communication content. Knowledge itself can also be run in the network system to promote the abundance of knowledge content, enhance the connotation of knowledge, obtain the kinetic energy required for location migration [43], and achieve the purpose of location transition. The position transition of knowledge network strengthens the intensity of knowledge, increases the activity of knowledge, improves the activity of knowledge field, breaks the original technical paradigm, creates new technical norms, and refreshes the technical practices of high-tech enterprises [44]. To sum up, put forward assumptions.

H5: knowledge network location transition positively regulates the impact of knowledge field activity and knowledge fermentation on technical inertia, respectively; that is, the higher the level of knowledge network location transition, the stronger the impact of knowledge field activity and knowledge fermentation on technical inertia.

### 2.4. Mediated Role

Hypothesis 2 and hypothesis 3 illustrate the intermediary role of knowledge field activity and knowledge fermentation, and hypothesis 4 expounds on the regulatory role of knowledge mobilization between the split fault of knowledge innovation network and technical practice. This study further infers that knowledge mobilization plays a regulatory role in the split fault of knowledge innovation network, and there is a regulated intermediary effect between the activity of knowledge field and knowledge fermentation on the whole intermediary mechanism of technological inertia. That is, knowledge mobilization contributes to the active transformation of the split fault of knowledge innovation network to technical practices through the activity of knowledge field and knowledge fermentation. Specifically, with the strengthening of the function of knowledge mobilization, the speed and accuracy of knowledge transfer among organizations will continue to improve. The split fault of knowledge innovation network provides more internal and external opportunities for knowledge mobilization so as to create an iterative update of knowledge system and improve the value performance of technical practices. On the contrary, knowledge mobilization is at a low level, and the integration efficiency of internal and external knowledge slows down. Even if the split fault of knowledge innovation network drives the operation mechanism of knowledge mobilization, the enterprise network organization system will still be unable to maintain continuous knowledge innovation and reduce the efficiency of technical practices due to the lack of effective control of operation.

Hypothesis 2 and hypothesis 3 illustrate the intermediary role of knowledge field activity and knowledge fermentation, and hypothesis 5 expounds on the regulatory role of knowledge network location transition between knowledge innovation network splitting fault and technical practice. This study further infers that the location transition of knowledge network plays a regulatory role in the whole intermediary mechanism of knowledge field activity and knowledge fermentation on technical inertia, and there is a regulated intermediary effect. That is, the location transition of knowledge network is conducive to the positive transformation of the split fault of knowledge innovation network to technical convention through knowledge field activity and knowledge fermentation. Specifically, with the strengthening of the location transition function of knowledge network, the speed and accuracy of knowledge transfer between organizations will continue to improve. The split fault of knowledge innovation network provides more internal and external opportunities for the location transition of knowledge network so as to create an iterative update of knowledge system and improve the value performance of technical practices. On the contrary, the position transition of knowledge network is at a low level, and the integration efficiency of internal and external knowledge slows down. Even if the split fault of knowledge innovation network drives the operation mechanism of knowledge network position transition, the enterprise network organization system will still be unable to maintain knowledge continuous innovation and reduce the efficiency of technical practices due to the lack of effective control of operation. Based on the above analysis, this study believes that knowledge mobilization and knowledge network location transition have a certain regulatory effect on the intermediary effect of knowledge innovation network split fault on technical practices through knowledge field activity and knowledge fermentation and puts forward hypotheses accordingly.

Hypothesis 6: knowledge mobilization and knowledge network location transition positively regulate the intermediary effect of knowledge innovation network splitting fault on technical practices through knowledge field activity; that is, the higher the level of knowledge mobilization, the stronger the intermediary effect of knowledge field activity.

Hypothesis 7: knowledge mobilization and knowledge network location transition positively regulate the intermediary effect of knowledge innovation network splitting fault on technical practices through knowledge fermentation; that is, the higher the level of knowledge network location transition, the stronger the intermediary effect of knowledge fermentation.

Based on the above analysis, this study believes that, in high-tech enterprises, the knowledge innovation network split fault can promote technical practice, and the knowledge field activity and knowledge fermentation have a certain media mechanism. The knowledge innovation network split fault further promotes enterprise technical practice through the intermediary role of knowledge field activity and knowledge fermentation, improving the innovation ability of high-tech enterprises. Knowledge mobilization and knowledge network location transition can regulate the activity of knowledge field and knowledge fermentation to a certain extent. It can adjust the intermediary medium, promote enterprise knowledge integration, reduce knowledge volatilization, and ensure the renewal toughness of enterprise knowledge. Accordingly, this study constructs a theoretical model of knowledge innovation network splitting fault, knowledge field activity, knowledge fermentation, knowledge mobilization, and knowledge network location transition relationship (as shown in Figure 3) and discusses the internal mechanism of the impact of knowledge innovation network splitting fault on enterprise technology practices.

#### 2.4.1. Data Source and Data Analysis

The sample data of this paper are from the eastern provinces and cities. The survey objects are the scientific and technological employees of high-tech enterprises. The data survey method of combining online and offline is adopted. In order to ensure the accuracy of the survey data and avoid the psychological hint effect of the questionnaire, the questionnaire was treated secretly, and the respondents were informed and treated about the issues related to anonymity and confidentiality before the survey. In order to ensure the achievement of the research purpose, 565 questionnaires were distributed, and 551 were recovered. Excluding 13 unqualified questionnaires, 538 valid questionnaires, the effective rate is 97.64%. According to the questionnaire data obtained from the survey, the characteristics of the survey samples are described in Table 1.

### 2.5. Variable Determination and Measurement

The scale used in problem analysis mainly draws lessons from the mature scale design at home and abroad. The Likert scale 7 subscale system is used for variable measurement, and the value range is in the range of 1–7. The larger the value, the higher the degree of approval and, on the contrary, the lower the degree of approval.

Referring to the scale design research of Jehn and Bezrukova, Thatche and Patel, and Heidl et al., this paper measures five items from two dimensions: organizational attribute and interorganizational connection [10, 45, 46].

The knowledge field activity scale draws on the relevant research results of Senoo et al. and Gan and Qi [20, 47]. The activity of knowledge field is measured by four items: “good cohesion among employees within the enterprise,” “smooth level of enterprise cooperation, interaction, and communication,” “strong active learning atmosphere,” and “enterprise personnel participating in external technical exchange and cooperation.”

The Knowledge Fermentation Scale refers to the research results of Wang and Liu and He [24, 48]. The measurement of knowledge fermentation is measured from four dimensions and six items: development direction, communication channel, academic thought, and management mechanism.

Based on the research of Yao et al., the Knowledge Mobilization Scale measures employee enthusiasm, employee communication, organizational cooperation, scientific research and innovation ability, organizational planning, and other aspects, with a total of 6 items [49]. Referring to the research of Paruchrui [50], the knowledge network location transition scale is composed of five items: the link members of enterprises in the network, the status of enterprises in the network, and the relationship with other enterprises from the two dimensions of network location centrality and network location intermediary.

The design of technical convention scale refers to the scale design research of Sun and Dang, Garca-Morales et al., Tatarynowicz et al., and so on [1, 51, 52]. This paper measures four items from the two dimensions of behavior tacit understanding and specification.

## 3. Empirical Analysis Results

### 3.1. Descriptive Statistical Analysis and Test

The relevant variables are statistically described, and the results are shown in Table 2. The Pearson correlation coefficients of different variables are between 0.5 and 0.7, indicating that there is a certain correlation between the variables.

### 3.2. Reliability and Validity Test of the Scale

The common method deviation involved in this paper is tested by controlling the nonmeasurable potential factor method. The new potential marker variable is set as knowledge filtering. Compared with the goodness of fit index corresponding to the structural equation model before control, the goodness of fit index of the structural equation model after control is relatively poor. The change amount of the main goodness of fit index is as follows: the absolute change amount corresponding to the ratio between chi-square and degree of freedom is 0.094, and the absolute change amount of the NFI index is 0.02. The absolute change of the IFI index is 0.02, the CFI index is 0.01, and the RMSEA index is 0.02, which further shows that there is no serious common variance deviation in this paper.

Cronbach's coefficient > 0.5 (Table 3), indicating that each variable has good reliability. Kmo test values are greater than 0.5, indicating that the variables have an excellent structural framework. The reliability CR of variable combination in the table is > 0.80, indicating that the reliability of design variable construction is good. Ave value is > 0.5, and the convergence validity of design variables is good.

### 3.3. Conceptual Model and Research Hypothesis Test

#### 3.3.1. Analysis and Test of the Main Effect of Knowledge Innovation Network Splitting Fault

According to the main effect test results of knowledge innovation network split fault in Table 4, the regression coefficient of knowledge innovation network split fault to technical convention *β* is 0.417, the P-test value is less than 0.05, and the lower and upper limits of interval estimation of regression coefficient are 0.307 and 0.527, respectively, indicating that the split fault of knowledge innovation network has a significant positive impact on technical practices. The split fault of knowledge innovation network can strengthen the order of knowledge, promote the coupling and optimization of knowledge genes, and improve the technical practices of high-tech enterprises.

#### 3.3.2. Analysis and Test of Intermediary Function of Knowledge Field Activity

Referring to the intermediary test methods of Wen et al., the bootstrap method is used to analyze and test the active intermediary effect of knowledge field [53]. The results are shown in Table 5.

The intermediary utility of knowledge field activity is tested by a three-step method.

Firstly, the relationship between knowledge network splitting fault and knowledge field activity is tested. According to model 1 in Table 5, it can be seen that knowledge innovation network splitting fault has a significant positive impact on knowledge field activity (*β* = 0.764; *p* < 0.05). Secondly, model 2 shows the impact of knowledge innovation network splitting fault on technology practice, and knowledge innovation network splitting fault has a significant positive impact on technology practice (*β* = 0.646; *p* < 0.05). Finally, model 3 adds the activity of knowledge field into the regression model. Comparing model 2 and model 3, the impact of knowledge innovation network splitting fault on technical practice is reduced from *β* = 0.646 (*p* < 0.05) and decreased to *β* = 0.299 (*p* < 0.05). The mediating role of knowledge field activity is more clearly shown in Table 6. The split fault of knowledge innovation network can have a positive effect on technical practices through knowledge field activity.

#### 3.3.3. Analysis and Test of Intermediary Effect of Knowledge Fermentation

Referring to the intermediary test methods of Wen et al., the bootstrap method is used to analyze and test the intermediary effect of knowledge fermentation [53]. The results are shown in Table 7.

The intermediary effect of knowledge fermentation was tested by three-step method.

Firstly, the relationship between knowledge innovation network fragmentation fault and knowledge fermentation is tested. According to model 1 in Table 5, it can be seen that knowledge innovation network fragmentation fault has a significant positive impact on technical practices (*β* = 0.551; *p* < 0.05). Secondly, model 2 shows the impact of knowledge innovation network split fault on technical practices. From the results, the knowledge innovation network split fault has a significant positive impact on technical practices (*β* = 0.646; *p* < 0.05). Finally, model 3 adds knowledge fermentation to the regression model. Comparing model 2 and model 3, the impact of knowledge innovation network splitting fault on technical practices is reduced from *β* = 0.646 (*p* < 0.05) and decreased to *β* = 0.345 (*p* < 0.05), and knowledge fermentation had a significant partial mediating effect. The intermediary role of knowledge fermentation is more clearly shown in Table 8. The split fault of knowledge innovation network can have a positive effect on technical practices through knowledge fermentation.

#### 3.3.4. Analysis and Test of the Regulatory Role of Knowledge Mobilization

Using Wen et al. and other regulatory action test methods for reference, the bootstrap method is used for test, and the results are shown in Table 9 [54]. According to model 1 in Table 9, knowledge mobilization and knowledge activity have a significant positive impact on technical practices (*β* = 0.385, *p* < 0.05; *β* = 0.312, *p* < 0.05; *β* = 0.054, *p* < 0.05), indicating that knowledge mobilization has a good regulatory effect on the activity of knowledge field.  Table 10 describes the effect of knowledge mobilization on the activity of knowledge field in different situations, which can provide enterprises with different options and promote the improvement of enterprise innovation ability. Model 2 shows that knowledge mobilization and knowledge fermentation have a significant positive impact on technical practices (*β* = 0.087, *p* < 0.05; *β* = 0.513, *p* < 0.05; *β* = 0.122, *p* < 0.05), indicating that knowledge mobilization has a good regulatory effect on knowledge fermentation.

#### 3.3.5. Analysis and Test of Position Transition Regulation of Knowledge Network

Based on the regulation effect method proposed by Wen et al., the position transition test of knowledge network is completed (Table 11) [54]. According to model 1 in Table 11, the knowledge network location transition and knowledge field activity have a significant positive impact on technical practices (*β* = 0.018, *p* < 0.05; *β* = 0.723, *p* < 0.05; *β* = 0.054, *p* < 0.05), indicating that the position transition of knowledge network has a good regulatory effect on the activity of knowledge field.  Table 12 describes the effect of knowledge network location transition on the activity of knowledge field in different situations, which can provide different options for high-tech enterprises and improve the innovation ability of high-tech enterprises. Model 2 shows that knowledge network location transition and knowledge fermentation have a significant positive impact on technical practices (*β* = 0.001, *p* < 0.05; *β* = 0.734, *p* < 0.05; *β* = 0.188, *p* < 0.05), indicating that the position transition of knowledge network has a good regulatory effect on knowledge fermentation.

#### 3.3.6. Analysis and Test of the Mediating Effect of the Regulation of the Activity of Knowledge Field

The bootstrap method was used to test the mediating effect of the regulation of knowledge field activity. According to the result model 1 in Table 13, the interaction product term of knowledge mobilization and knowledge field activity is significant (*β* = 0.044, *p* < 0.05), indicating that the intermediary role of knowledge field activity is regulated by knowledge mobilization and positively affects technical practices.  Table 14 shows that when the level of knowledge mobilization is high (one standard deviation above the mean), the mediation value of knowledge network splitting fault from knowledge field activity to technical practice is 0.193, the confidence interval is [0.116, 0.257], excluding 0, and the mediation effect is significant. When the level of knowledge mobilization is low, the mediating effect of knowledge network splitting fault from knowledge field activity to technical practice is 0.161, the confidence interval is [0.101, 0.231], excluding 0, and the mediating effect is significant. There was a significant difference between the intermediary indirect effect values at higher and lower levels of knowledge mobilization (*p* < 0.05, CI [0.114, 0.245]). It shows that when the level of knowledge mobilization is stronger, the intermediary role of knowledge field activity between knowledge network splitting fault and technical practice is significantly enhanced.

The bootstrap method was used to test the mediating effect of the regulation of knowledge field activity. According to the result model 2 in Table 13, the interactive product term of knowledge field activity and knowledge network location transition is significant (*β* = 0.048, *p* < 0.05), indicating that the intermediary effect of knowledge field activity is regulated by the position transition of knowledge network, which has a positive impact on technical practices.  Table 15 shows that when the transition level of knowledge network location is high (one standard deviation above the mean), the mediation value of knowledge network splitting fault from knowledge field activity to technical convention is 0.185, the confidence interval is [0.116, 0.257], excluding 0, and the mediation effect is significant. When the position transition level of knowledge network is low (one standard deviation below the mean), the mediation value of knowledge network splitting fault from knowledge field activity to technical convention is 0.160, the confidence interval is [0.114, 0.245], excluding 0, and the mediation effect is significant. There is a significant difference between the intermediary indirect effect values when the knowledge network location transition is high and low (*p* < 0.05, CI [0.101, 0.220]). It shows that when the position transition level of knowledge network is stronger, the intermediary role of knowledge field activity between knowledge network splitting fault and technical practice is significantly enhanced.

#### 3.3.7. Analysis and Test of the Mediating Role of Knowledge Fermentation Being Regulated

The bootstrap method was used to test the mediated effect of knowledge fermentation. According to the result model 1 in Table 16, the interactive product term of knowledge mobilization and knowledge fermentation is significant (*β* = 0.028, *p* < 0.05), indicating that the intermediary role of knowledge fermentation is regulated by knowledge mobilization and has a positive impact on technical practices.  Table 17 shows that when the level of knowledge mobilization is high (one standard deviation above the mean), the mediation value of knowledge network splitting fault from knowledge fermentation to technical practice is 0.118, the confidence interval is [0.057, 0.169], excluding 0, and the mediation effect is significant. When the level of knowledge mobilization is low, the mediating effect of knowledge network splitting fault from knowledge fermentation to technical practice is 0.1053, the confidence interval is [0.073, 0.168], excluding 0, and the mediating effect is significant. There was a significant difference between higher and lower levels of knowledge mobilization (*p* < 0.05, CI [0.084, 0.182]). It shows that when the level of knowledge mobilization is stronger, the intermediary role of knowledge fermentation between knowledge network splitting fault through knowledge field activity and technical practice is significantly enhanced.

The bootstrap method was used to test the mediated effect of knowledge fermentation. According to the result model 2 in Table 16, the interactive product term of knowledge fermentation and knowledge network location transition is significant (*β* = 0.011, *p* < 0.05), indicating that the intermediary role of knowledge fermentation is regulated by the position transition of knowledge network, which has a positive impact on technical practices.  Table 18 shows that when the transition level of knowledge network location is high (one standard deviation above the mean), the mediation value of knowledge network splitting fault from knowledge fermentation to technical convention is 0.110, the confidence interval is [0.057, 0.169], excluding 0, and the mediation effect is significant. When the position transition level of knowledge network is low (one standard deviation below the mean), the mediation value of knowledge network splitting fault from knowledge field activity to technical convention is 0.105, the confidence interval is [0.068, 0.160], excluding 0, and the mediation effect is significant. There was a significant difference between the intermediate indirect effect values when the knowledge network location transition was high and low (*p* < 0.05, CI [0.073, 0.160]). It shows that when the position transition level of knowledge network is stronger, the intermediary role of knowledge fermentation between knowledge network splitting fault and technical practice is significantly enhanced.

## 4. Conclusion and Discussion

### 4.1. Research Conclusion

Based on the perspective of knowledge innovation theory, taking the activity of knowledge field and knowledge fermentation as intermediary variables, this paper discusses the role and influence mechanism of knowledge innovation network splitting fault on the technical practices of high-tech enterprises under the action of regulatory variables, knowledge mobilization, and knowledge network location transition and obtains the following empirical analysis conclusions:

1. The split fault of knowledge innovation network has a significant positive impact on the technological practices of high-tech enterprises. Through the research on the split fault of knowledge innovation network and the technical practice of high-tech enterprises, the split fault of knowledge innovation network can help enterprises update and iterate knowledge and maintain lasting technological innovation.
2. Knowledge field activity and knowledge fermentation play a partial intermediary role between the split fault of knowledge innovation network and enterprise technology practice in high-tech enterprises. In the process of technological innovation of high-tech enterprises, paying attention to the exchange of knowledge and the precipitation of content knowledge can break through the original technical bottlenecks and barriers of enterprises, maintain the activity of knowledge, and stimulate the inherent activity of knowledge ontology.
3. Knowledge mobilization and knowledge network location transition have a significant positive regulatory effect on the activity of knowledge field and knowledge fermentation on the technical practices of high-tech enterprises. The essence of knowledge innovation is the process of continuous accumulation, variation, and upgrading of knowledge. The continuous enhancement of the activity of knowledge field, knowledge migration, and superposition needs to communicate with external environmental subjects to promote knowledge renewal, integration, and reconstruction. Knowledge mobilization and knowledge network location transition can continuously promote the process of knowledge integration, improve the quality of knowledge connotation, and achieve a breakthrough in the paradigm of knowledge itself; the technological practices of high-tech enterprises have been innovated and upgraded.
4. Knowledge mobilization and knowledge network location transition play a regulatory role in the activity of knowledge field and knowledge fermentation on the intermediary effect between the split fault of knowledge innovation network and the technical practice of high-tech enterprises and provide assistance for enhancing the innovation ability of high-tech enterprises.

### 4.2. Theoretical Significance

1. This paper extends the study of antecedent variables of technical practices.
2. Previous studies on antecedent variables of technical conventions mostly focused on the expression of single information, and there are few paths and mechanisms to obtain high-value knowledge information based on massive network data. This paper expounds the research on the antecedent variables of technological practices from a unified level and multiple perspectives and defines the impact mechanism of the split fault of knowledge innovation network on the technological practices of high-tech enterprises, further expanding the research on technical practices.
3. This study reveals the mediating effect of knowledge field activity and knowledge fermentation on the split fault of knowledge innovation network and technical practice.
4. However, under the split fault of knowledge innovation network, there are few studies on the impact of knowledge field activity and fermentation on knowledge renewal, migration, and iteration of high-tech enterprises, and the mechanism of knowledge field activity and knowledge fermentation on knowledge renewal of high-tech enterprises is ignored.
5. Through the regulation of knowledge mobilization and knowledge network location transition on knowledge field activity and knowledge fermentation on technical practices, this study clarifies the regulation function of knowledge mobilization and knowledge network location transition on knowledge field activity and knowledge fermentation.
6. This study expounds on the impact of knowledge innovation network split fault on technology practice through the regulated role of knowledge mobilization and knowledge network position transition in the activity of knowledge field and knowledge fermentation on the split fault of knowledge innovation network and the intermediary effect of technology practice of high-tech enterprises. It enriches the research results of the impact of knowledge innovation network splitting fault on technical practices.

### 4.3. Practical Significance

The research conclusion of this paper can promote the continuous improvement of the innovation ability of high-tech enterprises and has reference value for the practice and management of improving the competitiveness of high-tech enterprises, which is embodied in the following.

Firstly, the split fault of knowledge innovation network has a positive effect on the technical practice of high-tech enterprises and can improve the innovation ability of high-tech enterprises. The split fault of knowledge innovation network can provide organizations with advanced ideas of integration and optimization of internal knowledge, technology, patents, and other aspects of enterprises, improve the innovation mechanism of high-tech enterprises, give full play to the enthusiasm of employees of high-tech enterprises, and break through the initiative of the original paradigm of knowledge subjects.

Secondly, we should attach importance to the intermediary role of knowledge field activity and knowledge fermentation of high-tech enterprises in the split fault of knowledge innovation network on technological practices so as to enhance the technological innovation ability of high-tech enterprises.

Thirdly, highlight the regulatory role of knowledge mobilization and knowledge network location transition in the activity of knowledge field and knowledge fermentation in the technical practices of high-tech enterprises.

Finally, it pays attention to the regulated function of knowledge mobilization and knowledge network position transition in the activity of knowledge field and knowledge fermentation on the intermediary effect of knowledge network splitting fault and high-tech enterprise technology practice.

Under the background of knowledge renewal growing at a geometric rate, obtaining effective knowledge in the shortest time is an important part of the formation of the competitiveness of high-tech enterprises. The regulated function of knowledge mobilization and knowledge network position transition in the activity of knowledge field and the intermediary effect of knowledge fermentation on the split fault of knowledge network and the technical practice of high-tech enterprises can fully mobilize the orderly flow of internal knowledge of high-tech enterprises, promote knowledge upgrading and iteration, improve the innovation ability of high-tech enterprises, and promote the impact of knowledge network splitting fault on technology practice in high-tech enterprises.

### 4.4. Research Limitations and Prospects

Although the research conclusion has certain theoretical value and practical reference significance for the construction of enterprise high-tech innovation, there are still some deficiencies.

Firstly, the data used in this study are from the questionnaire. When the respondents fill in the questionnaire, the subjective preference of technicians is inevitable. In the future, the interview survey can be used to verify the data so as to improve the accuracy of the sample data as much as possible.

Secondly, the concept of knowledge innovation network split fault comes from the vocabulary in geography [55], but there is still room for further study on the definition of its connotation and dimension. In this paper, the innovation mechanism based on the thought of Technology Convention of high-tech enterprises is still in the development stage, the depth of research needs to be further excavated, and the research on the impact path and mechanism of Technology Convention is not perfect. It needs to be further studied to explore its impact on the innovation competitiveness of high-tech enterprises.

## Figures and Tables

**Figure 1:** Categories of knowledge innovation network split fault. (a) Transverse fault. (b) Longitudinal fault. (c) Oblique fault.

**Figure 2:** Knowledge fermentation model.

**Figure 3:** Research conceptual model 2 study design.

**Table 1:** Description of sample characteristics.

	Attribute	Quantity (proportion)
Region	Eastern region	538
Level	State owned and state holding	15
	Joint venture and private	26
Industry	High-tech industry	41
Years of establishment	Less than 5 years	18
	5–10 years	16
	More than 10 years	7
Enterprise scale	Less than 300 people	135
	300–1000 people	285
	More than 1000 people	118
Respondent position	Senior technicians	47.3%
	Middle level technicians	52.7%
Education background of respondents	Below bachelor's degree	282
	Bachelor's degree or above	256
Years of work investigated	Less than 5 years	142
	5–10 years	247
	More than 10 years	149
Investigated gender	Male	289
	Female	249

**Table 2:** Descriptive statistics and correlation coefficient.

	Mean	Std. deviation	B1	B2	B3	B4	B5	B6
Knowledge innovation network split fault	3.999	1.011	1.000					
Knowledge field activity	3.671	1.072	0.720^*∗∗*^	1.000				
Knowledge fermentation	3.723	0.944	0.591^*∗∗*^	0.621^*∗∗*^	1.000			
Knowledge mobilization	3.728	1.181	0.596^*∗∗∗*^	0.606^*∗∗*^	0.596^*∗∗*^	1.000		
Knowledge network position transition	3.900	0.991	0.602^*∗∗*^	0.621^*∗∗*^	0.617^*∗∗*^	0.644^*∗∗*^	1.000	
Technology practices	3.560	1.118	0.586^*∗∗*^	0.561^*∗∗*^	0.537^*∗∗*^	0.550^*∗∗*^	0.654^*∗∗*^	1.000

*Note.* ^*∗∗*^Significant at the level of 5%.

**Table 3:** Reliability and validity test of the scale.

	Number of items	Kmo value	Cronbach's coefficient	Factor load factor	CR	Ave
Knowledge innovation network split fault	5	0.501	0.677	0.513	0.841	0.519
				0.675		
				0.812		
				0.802		
				0.758		

Knowledge field activity	4	0.616	0.625	0.626	0.810	0.518
				0.704		
				0.817		
				0.719		

Knowledge fermentation	6	0.666	0.730	0.564	0.877	0.556
				0.473		
				0.675		
				0.827		
				0.922		
				0.897		

Knowledge mobilization	6	0.596	0.514	0.661	0.897	0.604
				0.464		
				0.886		
				0.878		
				0.701		
				0.961		

Knowledge network position transition	5	0.814	0.879	0.673	0.850	0.536
				0.814		
				0.813		
				0.539		
				0.782		

Technology practices	4	0.719	0.676	0.791	0.903	0.699
				0.780		
				0.866		
				0.902		

**Table 4:** Main effect test results of knowledge network splitting fault.

Main effect	Effect	se	t	*p*	LLCI	ULCI
Knowledge innovation network split fault	0.417	0.056	7.456	0.000	0.307	0.527

**Table 5:** Intermediary role of knowledge field activity.

	Model 1 dependent variable knowledge field activity	Model 2 dependent variable technology practices	Model 3 dependent variable technology practices
Knowledge innovation network split fault	0.764^*∗∗*^ (*t* = 23.162) (0.699, 0.828)	0.646^*∗∗*^ (*t* = 16.141) (0.567, 0.724)	0.417^*∗∗*^ (*t* = 7.46) (0.477, 1.119)
Knowledge field activity			0.299^*∗∗*^ (*t* = 5.68) (0.196, 0.403)

*Note.* (1) ^*∗∗*^Significant at the level of 5%. (2) The values in brackets are interval estimates.

**Table 6:** Knowledge field activity Mediating effect and confidence interval.

	Indirect effect estimation	95% confidence interval	
	(standardized)	Lower limit	Upper limit
Knowledge field activity	0.208	0.134	0.283

*Note.* (1) ^*∗∗*^Significant at the level of 5%. (2) The values in brackets are interval estimates.

**Table 7:** Intermediary role of knowledge fermentation.

	Model 1 dependent variable knowledge fermentation	Model 2 dependent variable technology practices	Model 3 dependent variable technology practices
Knowledge innovation network split fault	0.551^*∗∗*^ (*t* = 16.351) (0.485, 0.618)	0.646^*∗∗*^ (*t* = 16.141) (0.567, 0.724)	0.455^*∗∗*^ (*t* = 9.586) (0.362, 0.549)
Knowledge fermentation			0.345^*∗∗*^ (*t* = 6.784) (0.245, 0.445)

*Note.* (1) ^*∗∗*^Significant at the level of 5%. (2) The values in brackets are interval estimates.

**Table 8:** Knowledge fermentation mediating effect and confidence interval.

	Indirect effect estimation	95% confidence interval	
	(standardized)	Lower limit	Upper limit
Knowledge fermentation	0.173	0.112	0.234

**Table 9:** Regulating role of knowledge mobilization.

	Model 1 dependent variable technology practices	Model 2 dependent variable technology practices
Mediating variables Knowledge field activity Knowledge fermentation	0.385^*∗∗*^ (*t* = 8.338) (0.294, 0.475)	0.087^*∗∗*^ (*t* = 1.1357) (-0.063, 0.236)
Moderating variables Knowledge mobilization	0.312^*∗∗*^ (*t* = 7.477) (0.230, 0.394)	0.513^*∗∗*^ (*t* = 14.256) (0.442, 0.584)
Interactive product term Knowledge field activity*∗*knowledge mobilization Knowledge fermentation*∗*knowledge mobilization	0.054^*∗∗*^ (*t* = 2.047) (0.002, 0.105)	0.122^*∗∗*^ (*t* = 2.218) (0.032, 0.229)

*Note.* (1) ^*∗∗*^Significant at the level of 5%. (2) The values in brackets are interval estimates.

**Table 10:** Knowledge mobilization moderating effects and confidence interval.

Adjustment quantity	The moderating effects of knowledge mobilization on knowledge field activity			The moderating effects of knowledge mobilization on knowledge fermentation		
Adjustment intensity	Effect estimation	95% confidence interval		Effect estimation (standardized)	95% confidence interval	
	(standardized)	Lower limit	Upper limit		Lower limit	Upper limit
High	0.448^*∗∗*^ (*t* = 7.6559)	0.333	0.723	0.230	0.036	0.425
Middle	0.385^*∗∗*^ (*t* = 8.338)	0.294	0.475	0.087	0.063	0.236
Low	0.321^*∗∗*^ (*t* = 6.136)	0.219	0.424	0.057	0.141	0.255

*Note.* (1) ^*∗∗*^Significant at the level of 5%.

**Table 11:** Regulating effect of knowledge network position transition.

	Model 1 dependent variable technology practices	Model 2 dependent variable technology practices
Mediating variables Knowledge field activity	0.018^*∗*^ (*t* = 0.7415) (−0.031, 0.068)	
Knowledge fermentation		0.001^*∗∗∗*^ (*t* = 0.180) (−0.136, 0.139)
Moderating variables Knowledge network position transition	0.723^*∗∗*^ (*t* = 18.0023) (0.644, 0.802)	0.734^*∗∗*^ (*t* = 18.929) (0.658, 0.811)
Interactive product term Knowledge field activity^*∗*^knowledge network position transition	0.054^*∗∗*^ (*t* = 2.444) (0.011, 0.098)	
Knowledge fermentation^*∗*^knowledge network position transition		0.188^*∗∗*^ (*t* = 3.027) (0.066, 0.309)

*Note.* (1) ^*∗*^, ^*∗∗*^, ^*∗∗∗*^Significant at the level of 5%. (2) The values in brackets are interval estimates.

**Table 12:** The moderator effect of knowledge network position transition and confidence interval.

Adjustment intensity	Effect estimation (standardized)	95% confidence interval		Effect estimation (standardized)	95% confidence interval	
		Lower limit	Upper limit		Lower limit	Upper limit
High	0.072^*∗∗*^ (*t* = 2.041)	0.002	0.142	0.187^*∗∗*^(*t* = 2.246)	0.120	0.354
Middle	0.019^*∗∗*^ (*t* = 2.214)	0.031	0.068	0.089^*∗∗*^(*t* = 2.148)	0.136	0.239
Low	0.035^*∗∗*^ (*t* = 2.023)	0.027	0.096	0.185^*∗∗*^(*t* = 2.202)	0.113	0.382

*Note.* (1) ^*∗∗*^Significant at the level of 5%. (2) The values in brackets are interval estimates.

**Table 13:** Regulated mediators of knowledge field activity and their tests.

	Model 1 dependent variable technology practices	Model 2 dependent variable knowledge field activity	Model 3 dependent variable technology practices	Model 4 dependent variable knowledge field activity
Independent variable Knowledge innovation network split fault	0.417^*∗∗*^ (*t* = 7.457) (0.477, 0.527)	0.426^*∗∗∗*^ (*t* = 4.478) (0.240, 0.615)	0.417^*∗∗*^ (*t* = 7.457) (0.477, 0.527)	0.391^*∗∗∗*^ (*t* = 3.533) (0.137, 0.608)
Mediating variables Knowledge field activity	0.299^*∗*^ (*t* = 5.677) (0.196, 0.403)		0.299^*∗*^ (*t* = 5.677) (0.196, 0.403)	
Moderating variables Knowledge mobilization		0.080^*∗∗*^ (*t* = 3.826) (0.110, 0.270)		
Knowledge network position transition				0.129^*∗∗*^ (*t* = 3.130) (0.095, 0.352)
Interactive product term Knowledge field activity^*∗*^knowledge mobilization		0.044^*∗∗*^ (*t* = 2.870) (0.002, 0.090)		
Knowledge field activity^*∗*^knowledge network position transition				0.048^*∗∗*^ (*t* = 3.789) (0.005, 0.100)

*Note.* (1) ^*∗*^, ^*∗∗*^, ^*∗∗∗*^Significant at the level of 5%. (2) The values in brackets are interval estimates.

**Table 14:** Regulated mediation and its test (knowledge innovation network split fault⟶knowledge field activity⟶knowledge mobilization⟶technology practices).

Moderating variables	Indirect effect (standardized)	95% confidence interval	
		Lower limit	Upper limit
High (+IS.D)	0.193	0.124	0.269
Low (-IS.D)	0.177	0.114	0.245
Difference	0.161	0.101	0.231

**Table 15:** Regulated mediation and its test (knowledge innovation network split fault⟶knowledge field activity⟶knowledge network position transition⟶technology practices).

Moderating variables	Indirect effect (standardized)	95% confidence interval	
		Lower limit	Upper limit
High (+IS.D)	0.185	0.115	0.257
Low (-IS.D)	0.174	0.111	0.232
Difference	0.160	0.101	0.220

**Table 16:** Regulated intermediaries and their inspection.

	Model 1 dependent variable technology practices	Model 2 dependent variable knowledge fermentation	Model 3 dependent variable technology practices	Model 4 dependent variable knowledge fermentation
Independent variable Knowledge innovation network split fault	0.455^*∗∗*^ (*t* = 9.560) (0.362, 0.549)	0.447^*∗∗*^ (*t* = 4.674) (0.259, 0.634)	0.455^*∗∗*^ (*t* = 9.590) (0.3619, 0.5485)	0.364^*∗∗*^ (*t* = 3.303) (0.147, 0.580)
Mediating variables Knowledge fermentation	0.345^*∗∗*^ (*t* = 6.784) (0.245, 0.445)		0.345^*∗∗*^ (*t* = 6.784) (0.245, 0.445)	
Moderating variables Knowledge mobilization		0.413^*∗∗*^ (*t* = 4.2717) (0.223, 0.603)		
Knowledge network position transition				0.436^*∗∗*^ (*t* = 3.845) (0.213, 0.658)
Interactive product term Knowledge fermentation^*∗*^knowledge mobilization		0.028^*∗∗*^ (*t* = 2.2113) (0.018, 0.074)		
Knowledge fermentation^*∗*^knowledge network position transition				0.0110^*∗∗*^ (*t* = 3.42) (0.041, 0.063)

*Note.* (1) ^*∗∗*^Significant at the level of 5%. (2) The values in brackets are interval estimates.

**Table 17:** Regulated mediation and its test (knowledge innovation network split fault⟶knowledge fermentation⟶knowledge mobilization⟶technology practices).

Moderating variables	Indirect effect (standardized)	95% confidence interval	
		Lower limit	Upper limit
High (+IS.D)	0.118	0.048	0.171
Low (-IS.D)	0.105	0.073	0.168
Difference	0.130	0.084	0.182

*Note.* (1) ^*∗∗*^Significant at the level of 5%. (2) The values in brackets are interval estimates.

**Table 18:** Regulated mediation and its test (knowledge innovation network split fault⟶knowledge fermentation⟶knowledge network position transition⟶technology practices).

Moderating variables	Indirect effect (standardized)	95% confidence interval	
		Lower limit	Upper limit
High (+IS.D)	0.110	0.057	0.169
Low (-IS.D)	0.107	0.068	0.160
Difference	0.114	0.073	0.160

## Data Availability

The data used to support the findings of this study are available from the corresponding author upon request.
